# Research on the Mechanism of HMGB1 Regulating Autoimmune Encephalomyelitis by Regulating NF-*κ*B

**DOI:** 10.1155/2022/9900916

**Published:** 2022-04-11

**Authors:** Lijuan Liu, Jingtao Pang, Hui Yuan, Shengnu Qiu, Wei Zhang, Zhenzhu Shang, Xiaoting Liu

**Affiliations:** ^1^The Third Department of Neurology, People's Hospital of Gaomi, Weifang, China; ^2^Second Department of Encephalopathy, Weifang Hospital of Traditional Chinese Medicine, Weifang, China; ^3^Division of Biosciences, Faculty of Life Sciences, University College London, London, UK

## Abstract

**Background:**

Autoimmune encephalomyelitis is a clinical condition in which memory and cognition is affected badly and is also associated with lower levels of consciousness or even coma in worse scenarios. It is a noninfectious condition which involves immune oriented inflammation.

**Objective:**

The study's goal was to figure out what was causing the problem HMGB1 involved in regulating the autoimmune encephalomyelitis by regulating NF-*κ*B.

**Materials and Methods:**

The expressions of HMGB1, miR-129-5p, and TLR4/NF-*κ*B signalling pathway-related proteins were measured by qRT-PCR. To explore the differences among its control, models, and all groups, histopathology, immunohistochemistry, and immunofluorescence tests were performed.

**Results:**

According to the findings, miR-129-5p is in charge of suppressing HMGB1 production and inhibiting the TLR4/NF-*κ*B signalling pathway. On development of autoimmune encephalomyelitis, neurons in the hippocampus area got injured in the miR-129-5p inhibitors class. In the miR-129-5p inhibitor class, expression of miR-129-5p reduced and HMGB1 elevated, increasing neuronal inflammation and damage. Impairment in the hippocampus, on the either side, was shown to be reduced in HMGB1 shRNA, miR-129-5p mimics, and TLR4/NF-*κ*B classes.

**Conclusion:**

According to the study's findings, there is indeed a link among increased miR-129-5p and decreased HMGB1 expression and also suppression of the TLR4/NF-*κ*B signal transduction pathway in autoimmune encephalomyelitis in the miR-129-5p inhibitors group. As a result, we may assume the autoimmune disease illness has progressed once concentrations of HMGB1, TLR4/NF-*κ*B, and miR-129-5p have decreased.

## 1. Introduction

EAE (experimental autoimmune encephalomyelitis) is a CNS autoimmune illness that is utilized as a model for studying sclerosis and abnormalities in individuals [1]. New clinical therapies have elaborated the emergence of autoimmune encephalomyelitis on the basis of autoantibodies linked to the nervous tissues. Most patients who had a good outcome were promptly diagnosed and treated. Limbic encephalitis is a prominent feature in the clinical phenotypes of autoimmune encephalomyelitis–AEM. Other features are behavior changes, disabled cognition, and seizures. Combination of cerebellar symptoms, optic neuritis, brainstem linked lesions, and myelitis are reported largely.

Autoimmune encephalomyelitis is an inflammatory condition which is immune-mediated and leads to dysfunction in the CNS [2, 3]. A nonneoplastic condition is usually triggered by environmental or hereditary factors.

NF-*κ*B (nuclear factor-*κ*B) is a transcription factor which is responsible for regulating large array genes linked in various processes associated with the immune system and inflammatory responses [4]. The activation of NF-*κ*B factor is linked to two main signalling pathways which are canonical and noncanonical pathways. Eventhough both have different mechanisms, but both are crucial for regulation of the inflammatory and immune responses [5, 6]. miR-129-5p, which targets the high-mobility group box 1 protein (HMGB1), has been shown to reduce renal fibrosis, according to Li Y et al. (Li et al., 2015). miR-129-5p may play a crucial role in AE-related epilepsy by regulating the TLR4/NF-*κ*B signalling pathway and particularly targeting HMGB1, as indicated earlier. In this study, we consequently aimed to identify the mechanism of HMGB1 involved in regulating the autoimmune encephalomyelitis by regulating NF-*κ*B.

## 2. Objective of Study

This study looked at the role of microRNA-129-5p (miR-129-5p) in the progression of autoimmune encephalomyelitis. A rat paradigm was used to identify HMGB1 targeted via the TLR4/NF-*κ*B signal transduction pathway. The miR-129-5p expression and its association with inflammation, reduction of expression, apoptosis, reduction in proliferation, differentiation, and neuronal growth were evaluated.

## 3. Materials and Methods

### 3.1. Animal Selection

70 Wistar rats, aged 10–12 weeks, have been used in this investigation, which were acquired from China Medical University's animal facility (Shenyang, China). The Laboratory Animal Ethical Committee approved the results of the experiment. Furthermore, 10 rats were included in the control group, while other random selections were selected for the induction of autoimmune encephalomyelitis via the animal model. Prior to any study, animals were permitted to acclimatize in a quality cage and were assigned unbound access to food and water. Before any therapy or surgery, a thermostat of 22–24°C was preserved, as well as a 12-hour light/dark cycle. The international guidelines for defense and analysis of pain in the laboratory animals were followed strictly. In the experimental study, the animals were divided as given in Table 1.

### 3.2. Establishment of the Autoimmune Encephalomyelitis Model

Wistar rats selected for the diseased group were injected subcutaneously with 0.06 ml/100 g of antigen emulsion. In the region near pad of the rear foot, a needle was inserted at 2/3 different positions for every injection leading to formation of a small bump near the foot pad. At same time, 0.05 ml pertussis bacilli (from Beijing Institute of Microbiology and Epidemiology, China) was injected intradermally in the back region of the foot pad. The region of injection was disinfected with alcohol. Immunization procedure was performed twice with a gap period of 7 days.

The behavior of rats was assessed postsensitization in accordance with the 5 criteria method via a blind study [7]. Here, 0, no sign of clinical symptom; 1, tail tension disappearance, awkward walking; 2, rear limb (weak); 3, paralysis in rear limbs; 4, hind limb paralysis/forelimb paralysis or weak muscles; 5, dead or dying. In between, symptoms were labeled via ±0.05. In the experiments conducted for the autoimmune encephalomyelitis paradigm sick class, rats scoring in the region of 2-3 were included [7].

### 3.3. Obtaining Tissues from Animal Models

Sections from tissues were collected after 24 hours postestablishment of the autoimmune encephalomyelitis model. Rats from both groups were anesthetized using 3 ml/kg pentobarbital sodium. The chest walls of animals were cut thus exposing the heart open. Postthoracotomy, a canula was fit in for opening aorta via ventricle (left). Furthermore, cannula implementation was performed for draining blood with help of ophthalmic scissors. Washing of the vessels was done with help of 150 ml 0.9% NaCl solution. Animals were injected with 4% polyformaldehyde fixing solution i.v at 8–10 ml/min.

After 30 minutes of the process, the body turned stiff. Heads of the rats were decapitated and kept in 0.9% NaCl for 2.5 hours. A blunt dissection was done on the right brain to isolate tissues from the hippocampal region. The sections were kept in at −80°C for IHC, histopathology, Western blotting, and qRT-PCR.

### 3.4. Immunohistochemistry and Immunofluorescence Analysis

Immunohistochemical histochemistry (IHC) was performed for analysis of tissue segments obtained from hippocampal region of the brain. The sections were implanted in paraffin followed by slicing into 5 *μ*m wide slides. Furthermore, these sections were deparaffinized followed by the dehydration by implementing graded alcohols. These slices were incubated for duration of fifteen minutes in a portion of 3% hydrogen peroxide in an ambient temperature (room temperature approx. 20°C) and blocked for 30 minutes in bovine serum.

The staining of the slides was done overnight at 40°C using antibody against caspase-3 (Thermo Fisher, USA). After this process, these sliced sections were further incubated for peripheral antibodies (Thermo Fisher, USA). For duration of three minutes, the immune-reactive sections were stained using diaminobenzidine (DAB) as well as covered using a cover slip. Slides were analyzed under a light microscope (Leica Microsystems) with 20x and 100x magnification.

Immunofluorescent analysis was performed on sections obtained from hippocampus. Furthermore, these sections were cleansed using the phosphate buffer saline followed by fixing for fifteen minutes in 4% paraformaldehyde, followed by blocking the sections in 5% BSA at an ambient temperature for duration of sixty minutes. Incubation with primary antibodies caspase-3 (Thermo Fisher, USA) was done at a temperature of 4°C night. The immediate day followed the incubation of the solution using the peripheral antibodies (Sigma Aldrich). Imaging of the tissues was performed postfluorescent staining and also identification of biomarkers such as caspase, NeUN, BrdU, and GFAP.

### 3.5. Assay for miRNA Microarrays

RNA was extracted from sections of the brain with help of the RNA extraction kit (Lexogen) in complete accordance to protocols. RNA was then quantified using the NanoDrop 8000 spectrophotometer (Thermo Fisher Scientific, USA). A total of 250 ng RNA was labeled using fluorescent dye HY5 with help of the Qubit™ microRNA Assay Kit (Thermo Fisher Scientific, USA). The labelling kit and hybridization of LNA array was designed in basis of miRBase 22, which contained probes of mice, rats, and humans.

### 3.6. Implementing qRT-PCR

The isolated RNA accumulation was performed followed by reverse transcription implementing the TaqMan MicroRNA (ThermoFisher) Reverse Transcription kit. The reaction system was used with 15 *μ*l; the conditions were maintained at 16°C for 30 minutes, 42°C for 30 min, and 85°C at 5 min. Samples were added in 5 wells. 1 gRNA was employed to make cDNA, and *β*-actin was employed as an internal control. The 2-Ct technique was used to identify relative quantity. To acquire the overall average, each test was done.

The primer sequence for HMGB1 was forward: 5′-AAGGAGAACATCCTGGCCTGTC-3'; reverse: 5′-TCCCAGTTTCTTCGCAACATCA-3' and for NF-*κ*B was forward: 5′-GCATTCTGACCTTGCCTATCT-3′; reverse: 5′-CTCCAGTCTCCGAGTGAAGC-3'. These experiments were individually carried out in a triplicate order for a final average value [8].

### 3.7. Western Blotting

In the hippocampal tissues isolated from all groups, a through washing done by the PBS (phosphate buffer saline) group was done using protease inhibitor. The blend was shivered at a temperature of 4°C for duration of five minutes followed by centrifugation (12000 ×g) for around ten minutes at a temperature of 4°C. The collection of supernatant fluid is performed for the protein extraction. TLR4 (Abcam, rabbit polyclonal, ab150583) and NF-*κ*B (Abcam, rabbit monoclonal, ab32536) primary monoclonal antibodies were used to incubate the membrane overnight (1 : 1200).

### 3.8. Statistical Analysis

SPSS 21.0 (SPSS Inc., IL, USA) was the tool implemented for statistical analysis. The data were portrayed in terms of mean ± standard deviation. A comparative assessment between both groups was performed using the *t*-test. *P* < 0.05 was counted as statistically significant.

## 4. Results

According to the results of the experiments, the neurological injury (Figures 1–3) has been most commonly recorded in the miR-129-5p blocker class, where the neuronal in the rats' hippocampal were badly injured. In classes III, V, VI, VII, the miR-129-5p mimics group, HMGB1 shRNA, and miR-129-5p mimics + HMGB1 shRNA class, the damages were found to be minor.

In each of the seven experimental classes, the mRNA expression of miR-129-5p and HMGB1 was examined. The finding indicated that the outcomes of the controls and TLR4/NF-*κ*B classes were not significantly different (*P* > 0.05). The expressions of miR-129-5p in the miR-129-5p mimic + HMGB1 and miR-129-5p mimics classes, but at the other extreme, were higher than the control class (*P*0.05), as shown in Figure 4.

When compared to the control group and the model class, the detected expression of HMGB1 mRNA in the miR-129-5p mimics class, HMGB1 shRNA, and miR-129-5p mimics + HMGB1 shRNA class was statistically meaningful (all *P*0.05). The transcription of miR-129-5p was considerably lower in the miR-129-5p inhibitory league compared to the deterministic model (*P*0.05), whereas the expression of HMGB1mRNA was way greater in the miR-129-5p inhibitor class compared with the control group, prototype category (*P*0.05).

The expression of miR-129-5p and HMGB mRNA was shown to be inversely linked, with miR-129-5p overexpression suppressing the expression of HGMB1. The expression of mRNA HMGB1 was constant across all seven classes, according to Western blotting. The expression of HMGB1 was not substantially different in the control, TLR4/NF-*κ*B, and model groups (*P* > 0.05). When compared to the control, prototype category, HMGB1 expressions were observed to be lower in the miR-129-5p mimics group, shRNA group, and miR-129-5p mimics + HMGB1 shRNA class (*P*0.05) (Figure 5).

The mRNA expression of TLR4/NF-*κ*B related proteins was shown to be steady. The obtained expressions of proteins associated with the TLR4/NF-*κ*B signalling pathway were not statistically significant when *P*0.05 was used. There was a significant drop in TLR4/NF-*κ*B protein expression when miR-129-5p mimics, HMGB1 shRNA, and miR-129-5p mimics + HMGB1 shRNA classes were compared to the reference and model classes (*P* > 0.05) [9]. The miR-129-5p inhibitors class highly (*P*0.05) mirrored high levels of mRNA expressions of TLR4/NF-*κ*B associated proteins, as shown in Figure 6 [10], (Figure 7).

Dense fibers were noted in the miR-129-5p inhibitors class in contrast to the normal group which might be due to initial inflammation subjected to evolution of autoimmune encephalomyelitis.

BrdU: this marker was responsible for identification of the generation and proliferation of neuronal cells in both control and miR-129-5p inhibitor groups. It also denotes the neuroprogenitors emerging in the BrdU injection period thus helping in evaluation of inflammation and damage. The proliferation of new formed neurons was visualized by the process of immunostaining for the marker BrdU which identifies proliferation of neurons. Expressions of BrdU were higher in control groups in contrast with the miR-129-5p inhibitors class in the hippocampal sections; thus, it can be interpreted that the proliferation declined in miR-129-5p inhibitor class. Thus, the conclusion obtained signified the reduction in proliferation in experimental autoimmune encephalomyelitis.

Caspase: detection of dense caspase signifies of cell death via apoptosis. The domination of caspase was noted in the miR-129-5p inhibitor class, while caspase was found to be not significant in the control class. Hence, it was interpreted that inflammation due to EAE leads to early apoptosis in the hippocampal region of the brain.

NeUN: NeUN is marker for differentiation of neurons. It is mainly expressed in nuclei of most neurons. A decrease in NeUN was noted in the miR-129-5p inhibitor class, thereby signifying the degeneration as well as inflammation due to encephalomyelitis in hippocampal region of the brain.

GFAP: it is an astrocyte marker of the protein present in the neurons. In the control group, GFAP was found significant. The immune system addressed the glial fibrillary acidic proteins in the miR-129-5p inhibitor family, resulting in a decrease in their density.

## 5. Discussion

When compared to the control and model groups, the expression of TLR4/NF-*κ*B group signalling pathway-related proteins in the HMGB1 shRNA category, TLR4/NF-*κ*B group, miR-129-5p mimics group, and miR-129-5p mimics + HMGB1 shRNA group dropped, while those in the miR-129-5p inhibitors team elevated.

This study's preliminary findings confirmed the hypothesis that miR-129-5p expression improved in the miR-129-5p mimics and miR-129-5p mimics + HMGB1 shRNA groups when compared to the control and model groups. The levels of HMGB1 mRNA and protein expression in the HMGB1 shRNA, miR-129-5p mimics, and miR-129-5p mimics + HMGB1 shRNA groups, on the other hand, decreased. This revealed a negative relationship between miR-129-5p and HMGB1, as well as the possibility of miR-129-5p overexpression suppressing HMGB1 production.

HMGB1-induced stimulation of the TL4/NF-*κ*B signal transduction pathway has also been identified as a critical stimulator of the cellular response to neuronal damage in vitro and in vivo, according to a recent research study. Studies have extensively posited a role for the HMGB1-TLR4/NF-*κ*B interplay in enabling the neuroprotection in preclinical animals of seizures and further proposed that upregulation of HMGB1 was likely to be an intrinsic activator of the TLR4/NF-*κ*B signalling pathway, which may advantage the remedy of neurodegeneration as well as neuroinflammatory illnesses, which is line with the observations of our study [10, 11], (Wang et al., 2010).

## 6. Conclusion

The study concludes by claiming that there is compelling evidence that miR-129-5p expression suppresses the TLR4/NF-*κ*B signalling cascade and HMGB1 transcription, therefore inhibiting the progression of autoimmune encephalomyelitis. It was also discovered because when miR-129-5p is repressed, the levels of HMGB1 and TLR4/NF-*κ*kB are elevated, meaning that when miR-129-5p is suppressed, the levels of HMGB1 and TLR4/NF-*κ*B are elevated in autoimmune encephalomyelitis. This must be viewed as a feasible aim in generating new therapy alternatives and acquiring a better knowledge of the illness.

## Figures and Tables

**Figure 1:** Histopathological analysis of the hippocampal region sectioned from the control and miR-129-5p inhibitors class.

**Figure 2:** Immunofluorescent staining of the tissue section by antibodies for identification of biomarkers BrdU, NeUN, GFAP, and caspase.

**Figure 3:** Percentage of normal neurons among various regions of the hippocampus in rat brain.

**Figure 4:** miR-129-5p and HMGB1 mRNA expressions in all groups.

**Figure 5:** Comparative assessment of HMGB1 protein expressions in rats among all groups.

**Figure 6:** TLR4/NF-*κ*B signalling pathway-associated proteins expression in all groups.

**Figure 7:** Expressions of TLR4/NF-*κ*B signalling pathway-associated proteins semiquantified.

**Table 1:** Experimental design.

S. no.	Group number	Treatment type	Number of animals (*n*)
1	I	Control group	10
2	II	Model group	10
3	III	miR-129-5p mimic group	10
4	IV	miR-129-5p inhibitor	10
5	V	HMGB1 shRNA	10
6	VI	TLR4/NF-*κ*B group	10
7	VII	miR-129-5p mimics + HMGB1 shRNA group	10

## Data Availability

The data used to support the findings of this study are available from the corresponding author upon request.

## Abbreviations

NF-*κ*B: Nuclear factor-*κ*B
miR-129-5p: MicroRNA-129-5p
AE: Autoimmune encephalomyelitis
EAE: Experimental autoimmune encephalomyelitis
CNS: Central nervous system
Caspases: Cysteine-aspartic proteases
NeUN: Hexaribonucleotide binding protein-3
GFAP: Glial fibrillary acidic protein
HMGB1: High-mobility group box 1 protein.
